# PLK1 Is a Potential Prognostic Factor Associated with the Tumor Microenvironment in Lung Adenocarcinoma

**DOI:** 10.1155/2022/7848771

**Published:** 2022-07-30

**Authors:** Lina Wang, Man Gao, Dongjie Sun, Haitao Wu, Shuang Lv, Yulin Li, Lisha Li

**Affiliations:** ^1^The Key Laboratory of Pathobiology, Ministry of Education, Department of Pathology, College of Basic Medical Sciences, Jilin University, Changchun, Jilin, China; ^2^Pediatric Department of Respiration II, The First Hospital of Jilin University, Changchun, Jilin, China; ^3^Cancer Center of the First Hospital of Jilin University, Changchun, Jilin, China

## Abstract

More than 40% of lung cancers are lung adenocarcinoma (LUAD) worldwide. However, the prognosis of LUAD is poor for the lack of effective treatment methods. Our study identified PLK1 as a novel prognosis biomarker and treatment target for LUAD. Based on the Cancer Genome Atlas (TCGA) database, differentially expressed genes (DEGs) from 551 LUAD cases were analyzed for the Kyoto Encyclopedia of Genes and Genomes (KEGG) enrichment analysis. To explore the biological pathways and the tumor-infiltrating immune cells (TICs) using gene set variation analysis (GSVA) and the CIBERSORT, as well as to analyze DEGs, a protein-protein interaction (PPI) network and Cox regression analysis were performed. Validation of DEGs was achieved through quantitative real-time PCR (qPCR) and immunoblotting. DEGs associated with the cell cycle were sorted out. Cell cycle scores were positively correlated with age, clinical stages, and metastasis and negatively correlated with overall survival of LUAD patients. PPI and Cox analyses showed that PLK1 could be a prognostic factor for LUAD patients. CIBERSORT analysis revealed a positive correlation between the transcription level of PLK1 and the function of CD8+ and activated memory CD4+ T cells, as well as a negative correlation with activated natural killer cells. Furthermore, PLK1 overexpression increased immune cytotoxicity, as measured by the cytolytic activity score, IFN- score, and IFN- level. There is a strong correlation between PLK1 and key features of TICs, indicating its potential as a promising prognostic biomarker for LUAD.

## 1. Introduction

Lung cancer is the most commonly occurring solid tumor worldwide [1]. Among all lung cancer cases, 85% of cases are non-small cell lung carcinoma (NSCLC). NSCLC includes adenocarcinoma, squamous cell carcinoma, and large cell carcinoma. Among them, the percentage of lung adenocarcinoma (LUAD) accounts for over 66% of all NSCLC cases [2]. Despite recent developments in the multiple targeted treatments and new immunotherapies for LUAD, the 5-year prognosis of LUAD patients is still very poor [3]. Such a phenomenon is possibly caused by the early dissemination and metastasis of LUAD. Moreover, the mechanisms underlying the onset and development of LUAD are unclear. Meanwhile, how the tumor-infiltrating immune cells (TICs) interact with LUAD is also poorly understood.

Several LUAD progression-correlated genes were reported. Elevated expression of the p53-inducible gene 3 (PIG3) is correlated with the incidence of lymph node metastasis in LUAD patients. It has been demonstrated to promote the development of LUAD through the enhancement of FAK/Src/paxillin pathway activation [4]. Enolase 1 (ENO1) is a protein-coding gene for a glycolysis enzyme related to glucose metabolism. It is also demonstrated to enhance LUAD tumor development. Recent research suggests that circ-ENO1 silencing causes a decrease in glycolysis, inhibits cell proliferation, and promotes apoptosis by suppressing the transcription level of ENO1 in LUAD patients [5]. Also, low expression levels of the ATM interactor (ATMIN) gene are reported to be associated with LUAD. Heterozygous ATMIN deficiency promoted tumor growth and raised cancer grade in an animal study of LUAD, which suggests that ATMIN can help fight LUAD [6]. Moreover, Polo-like Kinase 1 (PLK1) has been previously demonstrated to correlate with poor prognosis for LUAD patients [7]. However, it is still not clear how the transcription level of PLK1 is associated with TICs.

As accumulating evidence suggests, TICs play vital roles in regulating malignancy and therapy outcomes of various cancers through modulation of the tumor microenvironment (TME) [8]. Specifically, features of immune cells are found to be reliable indicators of the treatment outcomes of patients [9, 10]. Tumor-infiltrating T cells are found in over half of patients with ovarian cancer. The presence of tumor-infiltrating T cells is also significantly correlated with a better 5-year prognosis in ovarian cancer [11]. A clinical follow-up study of triple-negative breast cancer (TNBC) indicates that a better prognosis is associated with a high CD8+ T cell number (over 14%) [12]. High tumor-infiltrating lymphocytes (TILs) levels are also associated with low histologic grades of tumors [13]. In LUAD, patients with high TILs are also found to have better prognostic predictions in both progression-free survival (PFS) and overall survival (OS) [14].

This study was aimed to demonstrate the differences in TICs between LUAD and healthy lung tissue, confirm the correlation between hub genes and TICs, and unveil the possible mechanism underlying the onset and development of LUAD. Workflow details of this study are listed in Figure 1.

## 2. Materials and Methods

### 2.1. DEGs Extraction

The LUAD patients' transcriptome RNA-sequencing data (HTSeqFPKM) were obtained from the Cancer Genome Atlas (TCGA) database (https://portal.gdc.cancer.gov/), which contained 497 samples from LUAD patients' lungs and 54 samples from normal lung tissue. We downloaded the gene expression profile for GSE31210 using the Gene Expression Omnibus (GEO) databank (http://www.ncbi.nlm.nih.gov/geo/), including 226 samples from LUAD patients and 20 normal samples. The R packages “edgeR” and “limma” were applied to identify DEGs in the TCGA dataset and normalize the GSE31210 matrix data, respectively. The cutoff criteria for DEGs were an adjusted *p* value < 0.05 and |logFC| > 2.

### 2.2. GSVA and KEGG Enrichment Analysis

The R packages “GSVA” and “clusterProfiler” were used fo rGSVA (|log*FC*| > 0.3 and adjusted *p* value < 0.05 set as cutoff criteria) and KEGG enrichment analysis (adjusted *p* value < 0.05 set as cutoff criteria), respectively. The “c2.cp.kegg.v7.1.symbols.gmt” dataset was downloaded from Molecular Signature Database (http://software.broadinstitute.org/gsea/msigdb/index.jsp) and served as the reference gene set.

### 2.3. PPI Network and Cox Regression Analysis

Protein-protein interaction (PPI) network analysis was carried out by Search Tool for the Retrieval of Interacting Genes database (STRING, https://string-db.org/) (cutoff value: combined score ≥ 0.4) and illustrated by Cytoscape (version 3.6.0, https://cytoscape.org/). The R package “survival” was applied for Cox regression analysis (*p* value < 0.001).

### 2.4. Survival and Correlation Analyses

For the estimation of OS and PFS of LUAD patients, the R packages survival and survminer were used. Our survival curves were generated using the Kaplan-Meier method (significance was set as the *p* value < 0.05). Subsequently, Kaplan-Meier Plotter (https://kmplot.com/analysis/) and Gene Expression Profiling Interactive Analysis (GEPIA) (http://gepia.cancer-pku.cn/) were conducted for survival analysis. The Pearson coefficient was applied for correlation analysis using SPSS 22.0.

### 2.5. Validation of Gene Expression

The TCGA dataset and GSE31210 profile were used to perform statistical analyses for the hub genes. A meta-analysis developed using the Oncomine database (https://www.oncomine.org) was conducted to identify the expression pattern of hub genes in normal lungs and LUAD. To illustrate the level of protein expression, we utilized the immunohistochemical results of corresponding genes from the Human Protein Atlas (HPA, https://www.proteinatlas.org). Meanwhile, quantitative real-time polymerase chain reaction (qRT-PCR) and western blot analysis were used to assess the mRNA and protein expression levels of certain genes.

### 2.6. Assessment of Immune Activity of the TME

In all samples of LUAD, the relative proportion of TICs was estimated using the CIBERSORT computational method. The R package “corrplot” was applied for plotting the heat map of correlations among TICs. The FPKM values of the TCGA dataset were converted to Transcript Per Million (TPM) values, and the immune cytolytic activity score (CAS) was then calculated as the geometric mean of the *GZMA* and *PRF1* expression in TPM. IFN-*γ* score was defined as the mean of *CD8A*, *GZMA*, *GZMB*, *IFN-γ*, *EOMES*, *CXCL9*, *CXCL10*, and *TBX21* expression in FPKM.

### 2.7. Cell Cultures

BEAS-2B cells are normal cells; H1299, H1975, A549, and PC-9 cells are cancer cells. All cells were from Shanghai Institute of biology, Chinese Academy of Sciences. All cell lines were cultured in high glucose DMEM medium supplemented with 10% FBS and 1% penicillin/streptomycin (37 °C, 5% CO2).

### 2.8. qRT-PCR

Total RNA Extraction Kits (Solarbo) were used for the preparation of total RNA. cDNA was produced by a first-strand cDNA synthesis kit (Invitrogen, USA). qRT-PCR was carried out on Applied Biosystems ABI PRISM 7300 plus platform. Primers for *PLK1* (Sense: 5′-AAAGAGATCCCGGAGGTCCTA-3′; Anti-sense: 5′-GGCTGCGGTGAATGGATATTTC-3′) and *GAPDH* (Sense: 5′-GGAGCGAGATCCCTCCAAAAT- ′; Anti-sense: 5′-GGCTGTTGTCATACTTCTCATGG-3′) were used.

### 2.9. Western Blotting Assay

After extraction of cell lysate and quantification of protein concentrations, 10% SDS-PAGE gels were used to separate proteins, and then they were transferred to 0.45 *μ*m PVDF membranes (ThermoFisher, Waltham, MA, USA). After blocking the membranes with 5% non-fat milk, the membranes were incubated with primary antibodies of PLK1 (Abcam, Cambridge, UK, dilute 1 : 1000, ab189139) and GAPDH (Abcam, dilute 1 : 1000, ab9485) at 4 °C overnight, followed by incubation with a horseradish peroxidase-conjugated secondary antibody (Bioss, Beijing, China) at room temperature for 1 hour and visualization on a Tanon 5200 (Tanon, Shanghai, China).

### 2.10. Statistical Analysis

The statistical analysis was conducted using R software (version 3.6.0) and SPSS (version 22.0). The correlation analysis was carried out via Pearson's correlation tests. Statistical differences in the Kaplan-Meier analysis were compared using the log-rank test. The student's *t*-test was used to analyze the qRT-PCR and western blotting results. We conducted all experiments at least three times, and a *p* value < 0.05 was deemed statistically significant.

## 3. Results

### 3.1. Upregulation of the Cell Cycle Pathway in LUAD

GSVA was conducted to explore KEGG pathways according to data extracted from the TCGA dataset. Compared with normal lung samples, a total of 48 KEGG pathways (19 downregulated and 29 upregulated) were significantly different in LUAD samples, as shown in Figure 2(a) and Supplementary Table S1, the patterns of which were visualized in a heat map, as shown in Figure 2(b). The 1,419 DEGs (310 downregulated and 1,109 upregulated) identified from the TCGA dataset were predominantly enriched in cell cycle, as shown in Figure 2(c), and ECM-receptor interaction, coagulation cascades, protein digestion and absorption, complement, and p53 signaling pathway, as shown in Figure 2(d) and Supplementary Table S2. The cell cycle was the only common pathway identified by GSVA and KEGG enrichment analyses, as shown in Figure 2(e).

### 3.2. Correlation of Cell Cycle Pathway with Overall Survival (OS) Rate and Clinical Characteristics in LUAD Patients

The TCGA dataset was analyzed further to determine if cell cycle pathway genes could be used as prognostic markers for LUAD patients. This analysis indicated higher cell cycle scores in LUAD samples than in normal samples (Supplementary Figure S1). The cell cycle score was significantly higher in males (*p* = 0.0036), N1-3 (*p* = 0.0007), and M1 (*p* = 0.0186) than in corresponding subgroups but not distinctively altered in age and T classification subgroups, as shown in Figures 3(a)to 3(e). Besides, cell cycle scores had a positive correlation with tumor stage in LUAD, as shown in Figures 3(f)and 3(g). The LUAD patients were categorized into high and low subgroups according to median cell cycle scores. Patient subgroups with high cell cycle scores had significantly worse OS and PFS, as shown in Figures 3(h) and 3(i).

### 3.3. Interaction Analysis of PPI Network and Univariate Cox Regression Analysis

A total number of 23 DEGs related to signaling pathways of the cell cycle were listed in Table 1. PPI network analysis was carried out using those DEGs and generated 23 nodes and 240 edges, as shown in Figure 4(a). The connectivity degrees of genes were estimated and illustrated in the histogram, as shown in Figure 4(b). In the results, DEGs including *BUB1B*, *CDC6*, *CDK1*, *MCM2*, *CDC20*, *CCNA2*, *CCNB1*, *CCNB2*, *CDC45*, *PLK1*, *CHEK1*, and *CCNE1* were found to have the highest degrees of connectivity. In addition, univariate Cox analysis showed that CCNA2, PTTG1, CDC25C, CCNB1, and PLK1 were associated with OS of LUAD patients, as shown in Figure 4(c). *CCNA2*, *CCNB1*, and *PLK1* were commonly found in the results of the PPI network (12 genes) univariate Cox analysis (5 genes), as shown in Figure 4(d).

### 3.4. High Expression of PLK1 in LUAD Samples

By comparing paired and unpaired difference analyses, PLK1 was significantly overexpressed in LUAD patients, as shown in Figures 5(a) and 5(b). In five different datasets, the meta-analysis revealed that PLK1 expression was significantly increased in the lung of patients with LUAD (Beer Lung [15], Garber Lung [16], Hou Lung [17], Stearman Lung [18], and Su Lung [19], as shown in Figure 5(c). According to immunohistochemical images obtained from HPA, PLK1 was expressed at a higher level in LUAD tissues than in normal tissues, as shown in Figure 5(d). Furthermore, we observed that PLK1 expression was significantly higher in LUAD than in normal lung tissues in the GSE31210 profile, as shown in Figure 5(e). Additionally, as validated by qRT-PCR and immunoblotting analysis, the transcription and protein levels of PLK1 were higher in H1975 and A549 cells than in BEAS cells, as shown in Figures 5(f) and 5(g).

### 3.5. Identification of PLK1 as a Prognostic Factor for the Patients with LUAD

Survival analysis and Cox regression analysis were carried out to evaluate *PLK1* as a prognostic marker. Our study found that high PLK1 expression was associated with poor overall survival in LUAD patients, as shown in Figures 6(a)to 6(c). The LUAD patients with high *PLK1* expression were negatively associated with PFS, as shown in Figures 6(d)to 6(f) . Meanwhile, the results of Cox analysis indicated that PLK1 might serve as an independent prognostic predictor for LUAD patients, as shown in Table 2. The *PLK1* expressive level was significantly increased in male versus female, T2-4 versus T1-2, N1-3 versus N0, and M1 versus M0 subgroups, as shown in Figures 7(a)to 7(d), but not in age subgroups, as shown in Supplementary Figure S2. Besides, PLK1 expressive level demonstrated a positive correlation with tumor stages in LUAD, as shown in Figures 7(e) and 7(f). LUAD patients were divided into two subgroups based on their median PLK1 expressive level. The high expression of PLK1 was significantly associated with poor OS, as shown in Figures 7(g)to 7(p) , and worse PFS (Supplementary Figure S3) in females, males, and T1-2, N0, M0, and stages I-II and stages III-IV subgroups, but not in T3-4, N1-3, and M1 subgroups.

### 3.6. Association of PLK1 with the Immune Activity of TME

To examine the relationship between PLK1 levels and the immune microenvironment of LUAD, TCGA datasets were analyzed, focusing on TICs, CAS, and IFN-*γ* scores. As shown in Supplementary Figure S4, CIBERSORT was used to estimate the fraction of 22 subtypes of immune cells that infiltrated the tumor. TIC profiles were visualized by the histogram. Meanwhile, the correlations between TICs were demonstrated in the heat map. A significant difference was found in the proportion scores of the 12 subtypes of TICs between high and low PLK1 level groups, as shown in Figure 8(a). Also, as revealed by the Pearson correlation analysis, 13 subtypes of TICs were significantly related to the PLK1 level, as shown in Figure 8(b). The 12 subtypes of TICs were commonly identified, as shown in Figure 8(c) and Supplementary Table S3. The generated results of changed TICs were identified as PLK1-associated TICs. In the results, the expressive levels of CAS and IFN-*γ* and scores of IFN-*γ* were increased in LUAD patients, as shown in Figures 9(a)to 9(c). Moreover, the expressive levels of CAS and IFN-*γ* and scores of IFN-*γ* were higher in LUAD patients with high PLK1 levels, as shown in Figures 9(d)to 9(f). Significant associations were found between the expressive levels of PLK1 and CAS, IFN-*γ*, and scores of IFN*-γ*, as shown in Figures 9(g)to 9(i).

## 4. Discussion

LUAD is one of the cancers with the highest mortalities. In the clinic, surgeries were the most widely used LUAD treatment method, mainly facilitated by early diagnosis. Combined surgery and chemotherapy resulted in an increase of 5-10% in survival [20]. However, the survival rates for LUAD patients are unsatisfactory. Poorly understood mechanisms related to the onset and development of LUAD also significantly limit the discoveries of novel effective treatment methods for LUAD patients. PLK1 was found to be a hub gene for cell proliferation in this study, which was positively correlated with clinical stages and cytotoxic activity in the TME.

PLK1 is known to participate in several cell cycle regulation pathways, including functioning as a G2/M checkpoint, participating in the regulation of centrosomes, spindle assemblies, and chromosome segregations [21]. Previous research found that a higher level of PLK1 was associated with malignant tumor incidence. Meanwhile, the overexpression of PLK1 negatively impacted the prognosis of patients with different types of cancers [22, 23]. Studies suggest that high PLK1 transcription and protein levels in gastric tumors are associated with a poor prognosis and treatment outcome [24]. A high PLK1 expression level was also strongly correlated with ovarian clear cell carcinoma (OCCC). In vitro, inhibition of PLK1 increased OCCC cell sensitivities to cisplatin treatments by enhancing autophagy and apoptosis [25]. A high expressive level of PLK1 was found to associate with TNBC according to a clinical study containing 3,173 samples. Overexpression of PLK1 significantly correlated to TICs and poor prognostic prediction of the patients. Gene set enrichment study found that genes related to cell cycle and MYC targets were significantly enriched in TNBC patients with high PLK1 expressive levels. A study *in vitro* has shown that PLK1 enhances the signaling of transforming growth factor (TGF)-*β* and therefore increases the invasiveness of cancer cells. This result was consistent with the clinical findings that the expression PLK1 robustly predicted the survival of patients with metastatic NSCLC [26]. Moreover, PLK1 was also suggested as a potentially effective treatment target for various types of cancer due to the suppressive effects on cell growth and promoting effects on apoptosis of tumor cells via the inhibition of PLK1 expression [27].

TICs have been successfully demonstrated to regulate the immune microenvironment of tumors and, therefore, impact the development of tumors and the treatment outcomes of cancer patients [28]. High tumor-infiltrating CD4+ and CD8+ T cell levels in pancreatic cancer strongly indicated a longer survival time [29]. Two subsets of tumor-infiltrating CD4+ and CD8+ T cells were found in NSCLC, respectively, expressing CD69 and CD103, both of which were markers of resident memory T cells [30]. Besides functioning as memory cells ready for quick responses to secondary infections, CD103+ T cells were also demonstrated to target tumor cells in previous studies [31]. Programmed cell death-1 (PD-1), CD244, and cytotoxic T-lymphocyte antigen-4 (CTLA-4) were majorly expressed on both CD8+ and CD4+ T cells.

Meanwhile, both tumor necrosis factor-alpha (TNF-*α*) and IFN-*γ* were predominantly produced by CD103+ CD4+ T cells [32–34]. Also, cytotoxic T cells were able to produce cytolytic effectors, including perforin (PRF1) and proapoptotic granzymes (GZMA), and participated in the immune reactions against tumor cells through the action of the granzyme-perforin pathway [35]. The results of previous studies have also indicated that CD56dim natural killer cells have dominant cytotoxic effects against tumor cells in a head and neck squamous cell carcinoma (HNSCC). In patients with HNSCC, it was found that CD56dim NK cells were associated with a promising prognosis [36]. Moreover, both infiltrating NK cells and macrophages indicated reasonable survival rates in patients with stage II and stage III esophageal cancer [37].

Most importantly, TME was demonstrated to substantially impact the cytotoxic effects of NK cells against tumor cells, possibly through its interaction with various signaling pathways related to the activation and infiltration of NK cells [38]. Moreover, the immune-regulatory effects mediated by TME were found in the suppression of infiltrating DCs in maintaining the homeostasis of CD8+ T cell immunoreaction and tumor antigen tolerance, leading to the promotion of tumor growth [39]. For this reason, the immune-regulatory effect of TME and the molecular mechanisms underlying this effect were proposed as pivotal factors in the development of new immunotherapy approaches for various cancers.

The findings of this study indicate that the expression level of PLK1 is related to clinical stages and the immune microenvironment of tumor cells. However, this study still contains some limitations. First, although qRT-PCR and western blotting were used to verify PLK1 expression in LUAD cell lines, the proposed mechanism of PLK1 regulation of tumor progression via the cell cycle needs further validation. Second, clinical samples were not used due to limitations on experimental conditions. Third, the correlation analyses of clinical characteristics were not satisfactory due to the unbalanced clinical data in the datasets. Finally, the association of PLK1 with TICs and molecular mechanisms was not fully elucidated.

## 5. Conclusions

This work represents a significant step forward in elucidating the molecular mechanisms behind LUAD progression. We discovered that *PLK1* might serve as a potential therapeutic target as well as a prognostic indicator for LUAD patients. *PLK1* is strongly correlated with several TICs in the tumor immune microenvironment. Further investigation should be conducted to improve the accuracy of the combined analysis and further illuminate the roles of PLK1 in the TIC community during LUAD progression.

## Figures and Tables

**Figure 1:** Flow chart for the PLK1 as a prognostic factor for lung adenocarcinoma (LUAD).

**Figure 2:** GSVA for samples and KEGG enrichment analysis for DEGs (a). 29 upregulated (red spots) and 19 downregulated (green spots) metabolic pathways were identified via GSVA in LUAD samples versus normal lung samples. Adjusted *p* value < 0.05 and |logFC| > 0.3 were utilized as the cutoff criteria for determining significant differences (b). Heat map for the significantly altered metabolic pathways (c). 1,109 upregulated (red spots) and 310 downregulated (green spots) DEGs were identified in LUAD samples versus normal lung samples. Adjusted *p* value < 0.05 and |logFC| > 2 were utilized as the cutoff criteria for determining significant differences (d). KEGG enrichment analysis for DEGs (e). Cell cycle was the common pathway identified in both GSVA and KEGG analyses.

**Figure 3:** Correlation of cell cycle score with clinical characteristics and survival of LUAD patients. The statistical difference for cell cycle score in LUAD patients with clinical traits, including age (a), gender (b), primary tumor (c), lymph node metastasis (d), distant metastasis classification (e), and tumor stage (f). The correlation of Cell Cycle scores with tumor stage (g). Kaplan-Meier curves for overall survival (OS) (h) and progression-free survival (PFS) (i) in high and low score patients grouped by the median of Cell Cycle score.

**Figure 4:** PPI network and univariate Cox analysis for the 23 DEGs in the cell cycle pathway (a). The PPI network consisted of 23 nodes (genes) and 240 edges (interactions between genes) (b). Histogram of the connectivity degrees of genes in the PPI network (c). Univariate Cox analysis for the 23 DEGs. A *p* value < 0.001 was utilized as the cutoff criterion (d). Venn diagram indicating 3 common genes which overlapped the 12 leading genes in the PPI network and the 5 prognosis-related genes in the Cox analysis.

**Figure 5:** Validation of PLK1 expression. PLK1 expression is significantly upregulated in LUAD samples compared to normal lung samples in both unpaired (a) and paired (b) difference analyses based on the TCGA dataset. PLK1 expression is significantly increased in LUAD samples compared with normal samples in a meta-analysis (c), immunohistochemical analysis (d), and GSE31210 profile (e). Gene expression level (f) and protein expression level (g) of PLK1 were significantly increased in H1975 and A549 cell lines compared with BEAS-2B cells. *n* = 3. Data represents mean ± SEM, ∗*p* < 0.05, ∗∗*p* < 0.01, ∗∗∗*p* < 0.001*vs.* BEAS-2B.

**Figure 6:** Correlation of PLK1 expression with the survival of LUAD patients. High *PLK1* expression is negatively associated with OS in LUAD according to TCGA dataset (a), GEPIA database (b) and Kaplan-Meier plotter platform (c). High *PLK1* expression predicted worse PFS relative to TCGA dataset (d), GEPIA database (e), and Kaplan-Meier plotter platform (f).

**Figure 7:** Prognostic significance of PLK1 in LUAD. The statistical difference for *PLK1* expression in LUAD patients with clinical traits, including gender (a), primary tumor (b), lymph node metastasis (c), distant metastasis classification (d), and tumor stage (e). The correlation of *PLK1* expression with tumor stage (f). Kaplan-Meier curves for the OS in LUAD subgroups with female (g), male (h), T1-2 (i), T3-4 (j), N0 (k), N1-3 (l), M0 (m), M1 (n), stages I-II (o), and stages III-IV (p).

**Figure 8:** Correlation of PLK1 expression with TICs proportion in LUAD patients. (a). Violin plot of the relative proportion of TICs in the high and low PLK1 expression subgroups grouped by median PLK1expression. Green-and red-colored columns represent the low and high PLK1 expression subgroups, respectively (b). Scatter plots for the significant correlation of the 13 TICs with PLK1 expression (c). Venn diagram indicating 12 kinds of common TICs overlapped by difference analyses and correlation tests.

**Figure 9:** Correlation of PLK1 expression with cytotoxic function. Histogram for cytolytic activity score (a), IFN-*γ* expression level (b), and IFN-*γ* score (c), which markedly increased in LUAD samples versus normal lung samples. Histogram for cytolytic activity score (d), IFN-*γ* expression level (e), and IFN-*γ* score (f) were significantly higher in the high PLK1 expression subgroup than the low PLK1expression subgroup. Values displayed were divided by median PLK1 expression. Scatter plots for cytolytic activity score (g), IFN-*γ* expression level (h), and IFN-*γ* score (i), which were significantly correlated with PLK1 expression.

**Table 1:** Differentially expressed genes in the cell cycle pathway.

Gene	logFC	*p* Value	Adjust *p* value
*CDC20*	3.681	8.76E-47	3.21E-45
*CDKN2A*	3.299	9.88E-19	8.65E-18
*CDC6*	3.140	4.56E-35	1.05E-33
*BUB1B*	3.042	2.42E-32	4.84E-31
*CCNE1*	3.000	1.78E-24	2.34E-23
*PLK1*	2.998	5.85E-37	1.45E-35
*CCNB1*	2.946	2.33E-44	7.85E-43
*CCNB2*	2.921	2.60E-37	6.54E-36
*CDC45*	2.894	2.51E-30	4.56E-29
*TTK*	2.849	1.96E-25	2.71E-24
*CDC25C*	2.811	9.20E-23	1.09E-21
*CCNA2*	2.791	4.82E-34	1.04E-32
*PKMYT1*	2.599	9.12E-26	1.29E-24
*ESPL1*	2.566	7.64E-21	7.91E-20
*ORC6*	2.528	1.12E-23	1.40E-22
*BUB1*	2.508	5.02E-28	8.14E-27
*ORC1*	2.431	6.50E-23	7.74E-22
*CDK1*	2.424	1.63E-30	3.01E-29
*MAD2L1*	2.384	2.76E-24	3.61E-23
*PTTG1*	2.305	3.80E-32	7.53E-31
*MCM4*	2.219	1.60E-37	4.05E-36
*CHEK1*	2.069	2.99E-22	3.41E-21
*MCM2*	2.014	2.82E-29	4.81E-28

Abbreviation: FC: fold change.

**Table 2:** Cox regression analysis for PLK1 expression on OS and PFS of LUAD patients.

Parameter	Univariate cox analysis			Multivariate cox analysis		
	HR	95% CI	*p* Value	HR	95% CI	*p* Value
TCGA (OS)						
Gender	1.035	0.717~1.495	0.852	0.927	0.638~1.347	0.691
Stage	1.654	1.401~1.951	<0.001	2.037	1.275~3.254	0.003
T classification	1.632	1.315~2.024	<0.001	1.189	0.940~1.503	0.149
M classification	1.757	0.964~3.203	0.066	0.353	0.103~1.210	0.098
N classification	1.790	1.459~2.196	<0.001	0.970	0.651~1.444	0.881
Age	1.002	0.983~1.021	0.843	1.013	0.993~1.033	0.192
*PLK1*	1.046	1.020~1.073	0.001	1.053	1.023~1.084	0.001
TCGA (PFS)						
Age	1.005	0.986~1.024	0.615	1.016	0.996~1.036	0.120
Gender	1.131	0.784~1.630	0.511	0.981	0.675~1.425	0.919
Stage	1.672	1.411~1.981	<0.001	1.575	1.031~2.405	0.036
T classification	1.573	1.285~1.926	<0.001	1.208	0.957~1.525	0.112
M classification	2.146	1.173~3.927	0.013	0.707	0.241~2.074	0.527
N classification	1.737	1.415~2.132	<0.001	1.130	0.789~1.619	0.505
*PLK1*	1.052	1.026~1.079	<0.001	1.057	1.028~1.086	<0.001
GSE31210 (OS)						
Age	1.025	0.977-1.075	0.306	1.035388	0.985-1.088	0.169
Gender	1.519	0.780-2.955	0.219	1.100991	0.547-2.215	0.787
Stage	4.232	2.175-8.236	<0.001	3.720136	1.886-7.337	<0.001
*PLK1*	1.658	1.192-2.306	0.003	1.538064	1.068-2.215	0.021

Abbreviations: LUAD: lung adenocarcinoma; HR: hazard ratio; CI: confidence interval; OS: overall survival; PFS: progression-free survival.

## Data Availability

This data can be found at The Cancer Genome Atlas database (https://cancergenome.nih.gov/), and Gene Expression Omnibus database (https://www.ncbi.nlm.nih.gov/geo/).

## Supplementary Materials

Supplementary Materials Supplementary Figure S1. Correlation of cell cycle score with LUAD patients. Supplementary Figure S2. Correlation of PLK1 expressive level with age subgroups of LUAD patients. Supplementary Figure S3. Correlation of high PLK1 expressive level with PFS of LUAD patients. Supplementary Figure S4. Correlation of PLK1 expression with tumor-infiltrating immune cells (TICs) in LUAD patients. Supplementary Table S1. Significantly changed metabolic pathways between LUAD and normal lung tissues. Supplementary Table S2. KEGG enrichment analysis for the DEGs. Supplementary Table S3. Immune cells significantly associated with PLK1 expression.
